The article "Yield improvement of exopolysaccharides by screening of the Lactobacillus acidophilus ATCC and optimization of the fermentation and extraction conditions" was published in 2016. Journal: EXCLI J.

# Yield improvement of exopolysaccharides by screening of the Lactobacillus acidophilus ATCC and optimization of the fermentation and extraction conditions

**DOI:** 10.17179/excli2015-356

**Published:** 2016-02-12

**Authors:** Qi Liu, Xingjian Huang, Dengxiang Yang, Tianlei Si, Siyi Pan, Fang Yang

**Affiliations:** 1 Department of Biological Engineering, Hubei University Zhixing College, Wuhan 430011, China; 2 College of Food Science and Technology, Huazhong Agricultural University, Wuhan 430070, China; 3 Key Laboratory of Environment Correlative Dietology (Huazhong Agricultural University), Ministry of Education, Wuhan, 430070, China; 4 Colloge of Animal Science and Technology, Huazhong Agricultural University, Wuhan 430070, China; 5 Key Laboratory for Green Chemical Process of Ministry of Education, Wuhan Institute of Technology, Wuhan 430073, China

**Keywords:** Plackett-Burman design, central composite design, EPS, fermentation optimization, extraction optimization

## Abstract

Exopolysacharides (EPS) produced by *Lactobacillus acidophilus *play an important role in food processing with its well-recognized antioxidant activity. In this study, a *L. acidophilus* mutant strain with high-yielding EPS (2.92±0.05 g/L) was screened by chemical mutation (0.2 % diethyl sulfate). Plackett-Burman (PB) design and response surface methodology (RSM) were applied to optimize the EPS fermentation parameters and central composite design (CCD) was used to optimize the EPS extraction parameters. A strain with high-yielding EPS was screened. It was revealed that three parameters (Tween 80, dipotassium hydrogen phosphate and trisodium citrate) had significant influence (P < 0.05) on the EPS yield. The optimal culture conditions for EPS production were: Tween 80 0.6 mL, dipotassium hydrogen phosphate 3.6 g and trisodium citrate 4.1 g (with culture volume of 1 L). In these conditions, the maximum EPS yield was 3.96±0.08 g/L. The optimal extraction conditions analyzed by CCD were: alcohol concentration 70 %, the ratio of material to liquid (M/L ratio) 1:3.6 and the extraction time 31 h. In these conditions, the maximum EPS extraction yield was 1.48±0.23 g/L. It was confirmed by the verification experiments that the EPS yield from *L. acidophilus* mutant strains reached 5.12±0.73 g/L under the optimized fermentation and extraction conditions, which was 3.8 times higher than that of the control (1.05±0.06 g/L). The results indicated that the strain screening with high-yielding EPS was successful and the optimized fermentation and extraction conditions significantly enhanced EPS yield. It was efficient and industrially promising.

## Introduction

Lactic acid bacteria (LAB), used for food fermentation since ancient times, currently has the “Qualified Presumption of Safety” (QPS) status for their long history of safe use in human consumption (EFSA, 2007[11]). Nowadays, many researches are concerned about the function of LAB for human's health such as preventing the diarrhea of children (Binns and Lee, 2010[4]), balancing the intestinal microecology (Lazado et al., 2011[24]), stimulating immunization (Johnson et al., 2012[21]; Perdigon et al., 1995[32]), removing the cholesterol (Liong and Shah, 2005[27]; Taranto et al., 1998[45]) and so on. Some of these functions are related to the EPS produced by LAB. 

The article "Yield improvement of exopolysaccharides by screening of the Lactobacillus acidophilus ATCC and optimization of the fermentation and extraction conditions" was published in 2016. Journal: EXCLI J.

EPS produced by LAB are long-chain polysaccharides consisting of branched, repeating units of sugars or sugar derivatives (Ismail and Nampoothiri, 2010[20]). It has been confirmed that EPS from LAB had most valuable application in the improvement of the rheology, texture and “mouth feel” of fermented milk products (German et al., 1999[16]; Vuyst et al., 2001[46]). Moreover, the EPS have been demonstrated to be antioxidant, antiulcer and antitumor with the ability to enhance the immune system as well as to lower blood cholesterol (Li et al., 2012[25]; Ruas-Madiedo et al., 2006[38], 2002[39]). Therefore, the EPS from LAB would be good bio-ingredients in food industry. 

However, all of these functions are affected by their chemical composition, molecular weight, electrical charge, the presence of lateral chains and the rigidity of EPS and they are also affected by the fermentation conditions and strain applied (Sánchez et al., 2006[43]). EPS produced by different strains vary in sugar composition, chain length, degree of branching, or sugar linkages under different fermentation conditions. Nevertheless, all these factors determine the rheological and health-promoting properties of EPS (Paturi et al., 2010[31]; Ruas-Madiedo et al., 2002[40]; Ruijssenaars et al., 2000[42]). There are two strategies for obtaining more EPS from LAB. In the first strategy, the high-yielding mutant strains should be obtained by chemical mutation or genetic engineering. And the other strategy is that the yield of EPS produced by LAB should be promoted by the optimization of fermentation conditions such as fermentation temperature, pH, the composition of cultural medium and so on (Årsköld et al., 2007[1]).

*L. acidophilus* is a safe bacterium and has been included in a variety of dairy products as a probiotic bacterium and its positive effects on human health have been indicated (Paturi et al., 2010[31]). However, there are only a few articles presenting the yield promotion of the EPS produced by *L. acidophilus* through chemical mutation or the fermentation condition optimization. In this paper, the high-yielding EPS-producing strain was obtained by chemical methods. Sixteen fermentation factors which may affect the yield of EPS produced by *L. acidophilus* were investigated by Placket-Burman (PB) and response surface methodology (RSM). Their main effects on EPS production and relative equations were quantified. Extraction parameters were optimized by central composite design (CCD). A novel strain with high-yielding EPS was obtained and the purpose of this essay was to promote the yield of EPS from* L. acidophilus* by screening the mutant strains and optimizing the fermentation parameters as well as extraction conditions for industrial application.

The article "Yield improvement of exopolysaccharides by screening of the Lactobacillus acidophilus ATCC and optimization of the fermentation and extraction conditions" was published in 2016. Journal: EXCLI J.

## Materials and Methods

### Strains and activation conditions

*L. acidophilus* ATCC used in this study as initial strain was obtained from the Institute of Microbiology, Chinese Academy of Science (Beijing, China). The initial strains were stored at -80 °C and incubated at 37 °C for 24 h in MRS broth for activation.

### EPS extraction and determination of the control

The activated initial strains were incubated in 30 mL MRS broth at 37 °C for 24 h. The cultures were centrifuged at 10000g/min for 30 min (Beckman, USA) and the precipitation was discarded. Alcohol (70 %, v/v) was added into the supernatants at 4 °C for 24 h to precipitate EPS and the ratio of the supernatants to 70 % alcohol (M/L ratio) was 1:3. The mixtures were centrifuged at 10000 g/min for 30 min, the precipitates were dissolved in 10 mL distilled water for quantitative determination of EPS with the phenol-sulfuric acid method using glucose as standard (DuBois et al., 1956[10]; Montersino et al., 2008[30]). These conditions were conducted as the control.

### Screening for high-yielding strains

The activated initial strains were cultivated in the MRS agar plates with 0.2 % diethyl sulfate. The mutant strains and the initial strains were vaccinated in the milk (100 mL) and the viscosities of the fermented milk were determined by digital viscometer (NDJ9s, Changzhou nuoji instrument, China) for the preliminary screening. 

The strains with the high viscosity of milk in the preliminary screening were incubated in the MRS broth medium (30 mL) at 37 °C for 24 h. EPS was extracted and determined as the method described in chapter “EPS extraction and determination of the control” and the high-yielding strains were selected according to the amount of the EPS.

### The optimization of fermentation condition for L. acidophilus ATCC

The 16 factors related to fermentation of the activated initial strains (presented in Table 1(Tab. 1)) were analyzed by PB experiments for choosing the most important influencing factors (Banik et al., 2007[3]). The variables, which were significant at 5 % level (P < 0.05) in the regression analysis, were considered to have greater impact on EPS yield and were further optimized by the steepest ascent experiment design and RSM. The content of the selected factors was determined by the steepest ascent experiment (Chen et al., 2009[9]; He and Tan, 2006[19]). 

The article "Yield improvement of exopolysaccharides by screening of the Lactobacillus acidophilus ATCC and optimization of the fermentation and extraction conditions" was published in 2016. Journal: EXCLI J.

Finally, the three critical factors affecting the fermentation of the activated initial strains were optimized by RSM (Box and Behnken, 1960[5]). The EPS yield was fitted by a second order model in order to correlate the response variable to the independent variables. The general form of the second degree polynomial equation is as follows [Equation 1]:

Y_i_= b_0_+ b_i_∑Xi +b_ii_∑X_i_^2^+b_ij_∑∑X_i_X_j _ [1]

In this formula, Y_i_ represented the content of EPS; X_i_, X_j_ represented the input variables; b_0_ represented the offset term; b_i _was the linear coefficient of X_i_; b_ii _was the quadratic coefficient of X_ii_ and b_ij _was the interaction coefficient. The experimental design was represented in Table 2(Tab. 2). 

### The optimization of extraction of EPS produced by L. acidophilus ATCC in MRS broth

The optimum ranges of the three factors (alcohol concentration, M/L ratio, and extraction time), which affected the extraction of EPS, were identified by signal factor experiments for the further optimization by CCD. The different alcohol concentrations (50 %, 60 %, 70 %, 80 %, and 95 %), M/L ratios (1:1, 1:2, 1:3, 1:4, and 1:5) and extraction times (6 h, 12 h, 24 h, 36 h, and 48 h) were operated in the signal factor experiments respectively. In each single factor experiment, one factor was changed while the other factors remained constant. The design matrix of the variables in coded units was presented in Table 3(Tab. 3). The model equation for analysis is as the same as Equation 1.

### Verification experiments

The EPS yields produced by the *L. acidophilus *ATCC mutant strains under the optimized fermentation and extraction conditions above were determined by the phenol-sulfuric acid method that was described in chapter “EPS extraction and determination of the control”. 

### Statistical analysis

All experiments were replicated three times (*n *= 3). Data from all replications each with triplicate analyses were analyzed using MINITAB 16 statistical software package (Minitab Inc., Pennsylvania, USA).

## Results and Discussion

### The obtaining of high yield mutation of L. acidophilus 

54 mutant strains were obtained by 0.2 % diethyl sulfate and the viscosity of the milk fermented by the 54 mutant strains was determined and the results were shown in Figure 1(Fig. 1). It showed that there was no significant difference between the viscosities of milk fermented by 8 mutations (No. 17, No. 18, No. 19, No. 27, No. 28, No. 31, No. 32, and No. 34) and that of initial strains (P > 0.05). Among the other mutations, the viscosity of milk fermented with 19 mutant strains rose significantly compared with that of initial strains (P < 0.05), while the other 27 mutant strains decreased the viscosity of milk significantly (P < 0.05). The highest viscosity of the fermented milk was 3303.3±17.5 mp·s.

The article "Yield improvement of exopolysaccharides by screening of the Lactobacillus acidophilus ATCC and optimization of the fermentation and extraction conditions" was published in 2016. Journal: EXCLI J.

The EPS yield of initial strain (control) was 1.05±0.06 g/L (Table 4(Tab. 4)), and the EPS yields of the 19 mutant strains that could increase the milk viscosity significantly were determined to gain the high-yielding mutant strains. Since the EPS yield of the No. 48 strains (2.92±0.05 g/L) was definitely higher than that of the other strains (P < 0.01), they were selected for the objection strain. 

Polysaccharide content is determined by anthrone colorimetry or phenol-sulfuric acid method with the wavelength at 620 nm or 490 nm (Southgate, 1976[44]). Therefore, we can screen the high EPS yield mutation through determining the polysaccharide content. However this operation is very complex and time-consuming. Some researchers have confirmed that the rheology of fermentation broths was generally attributed to the increasing polymer content (i.e., polysaccharide) (Bueno and Caracia-Cruz, 2001[6]; Philippis et al., 1991[33]). Also, there are some researches documenting that the polysaccharides from LAB contribute to the rheology, mouthfeel and texture of fermented milks, cheese or baked products (Galle et al., 2012[12]; Hamet et al., 2015[18]; Kristo et al., 2011[22]; Renard et al., 2006[36]). The reason may be that the EPS induces the interaction of the proteins to form protein bridges by combining peptides with water molecules on protein surface (Ayala-Hernandes et al., 2009[2]; Gentes et al., 2011[15]; Girard and Schaffer-Lequart, 2008[17]). Therefore, the rheology of fermented milk can be used to screen the high EPS yield mutation of *L. acidophilus* in the preliminary screening of the present study to simplify the experimental operation. The results also demonstrate that this method is feasible for high EPS yield mutation screening. 

### Screening fermentation conditions for high-yield EPS-producing strain with PB and RSM

The design matrix was selected to screen significant variables for the fermentation process of EPS and the corresponding results were shown in Table 1(Tab. 1). The coefficient of determination (R^2^) of the model was 0.990, which indicated that the model could explain 99.0 % of the data variation. The statistically significant effects of the variables were presented in Figure 2a(Fig. 2). Among the 16 fermentation variables, 7 variables (Dipotassium hydrogen phosphate, Tween 80, Trisodium citrate, Glucose, pH, Rotaton speed, Yeast extract) had statistically significant effect on the EPS yield (P < 0.05, significant at 5 % level) and the results were obtained from regression analysis. In the 16 variables, 6 variables had a positive influence on the EPS yield, while 6 variables had a negative effect on the EPS yield (Figure 2b(Fig. 2)). Among the 16 variables, Dipotassium hydrogen phosphate with a P value of 0.003 was identified to be the most significant factor, followed by Tween 80 (P = 0.004) and Trisodium citrate (P = 0.008). The lower P values indicated the more significant factors on the EPS yield. In the 3 factors, Tween 80 exerted a negative effect on the EPS yield, whereas the other two factors showed a positive influence on the EPS yield. Most bacteria can produce EPS under certain conditions, but the quantities and the composition of EPS are strain dependence and affected by the nutritional and environmental conditions. So it is possible to increase the polymer production by manipulating the culture conditions (Looijesteijn and Hugenholtz, 1999[28]; Xu et al., 2010[50]). The Plackett-Burman experiments can screen out main factors from a large number of process variables quickly, which are quite useful in preliminary studies and its principal objective is to select variables and their levels for further optimization processes (Reddy et al., 2008[35]). In the previous articles, 3 to 5 culture factors with most significant effect are selected (Chen et al., 2005[8]; Yasser et al., 2005[52]) or the factors with confidence interval from 80 % to 85 % are selected with Placket-Burman experiments for further optimization (Pujari and Chandra, 2000[34]; Xiong et al., 2004[49]). In the present study, 16 variables were selected to optimize polysaccharide fermentation conditions with Placket-Burman experiments and the three chosen variables with confidence interval above 95 % indicated that the further optimization would be more accurate. In the previous studies, medium components, inoculum size, fermentation time and temperature are determined as the significant factors in fermentation process by analyzing with PB experiments (Reddy et al., 2008[35]; Xu et al., 2010[50]). The results of this study revealed that the main impact factors for EPS produced by* L. acidophilus* were medium components (Trisodium citrate, Dipotassium hydrogen phosphate and Tween 80).

The article "Yield improvement of exopolysaccharides by screening of the Lactobacillus acidophilus ATCC and optimization of the fermentation and extraction conditions" was published in 2016. Journal: EXCLI J.

The optimum concentrations of the 3 variables determined by PB experiments were identified via the steepest ascent experiment. The design of the steepest ascent experiment is presented in Table 5(Tab. 5), and the results showed that the EPS yield of *L. acidophilus* initial strain rose at the beginning and then declined when the condition was that Tween 80 was 0.58 mL, Dipotassium hydrogen phosphate was 3.38 g, and Trisodium citrate was 3.14 g (Table 6(Tab. 6)). The highest EPS yield of *L. acidophilus* initial strain in the steepest ascent experiment was 3.59±0.05 g/L. Therefore, the corresponding conditions (Tween 80 0.58 mL, Dipotassium hydrogen phosphate 3.38 g, Trisodium citrate 3.14 g.) were collected for the further RSM. 

A quadratic model was constructed according to the data of 15 trials shown in Table 2(Tab. 2). By applying multiple regression analysis on the experimental data, second-order polynomial equation was found to explain the EPS yield of *L. acidophilus*. The mathematical model is as follows [Equation 2]:

Y=3.580-0.249X_1_+0.239X_2_+0.663X_3_-0.564X_1_^2^- 0.759X_2_^2^-0.271X_3_^2^+0.003X_1_X_2_+0.180X_1_X_3_+ 0.150X_2_X_3_. [2]

The results of ANOVA showed that F-value of regression was 76.90 (P < 0.01) and the F-value for lack of fit was 8.63 (P = 0.109), which indicated that the model is a good fit. The regression equation obtained from the ANOVA showed that the R^2^ was 0.983, which indicated that the model is capable of explaining 98.3 % of the variation in response. The R_adj_^2^ and R_pre_^2^ was 0.980 and 0.893 respectively and it had a good statistical model. The analysis results also indicated that Tween 80 had a significant negative effect on EPS yield and the other two factors had significant positive effect on EPS yield. The 3 factors showed significant negative quadratic effects on EPS yield (P < 0.01), indicating that EPS yields would decrease with the increase of the concentrations of these 3 factors. The interactions between the 3 factors above were also significant as results of the low P values (P < 0.01).

Figure 3(Fig. 3) showed the contour plots of EPS yield for each pair of nutrient concentration by keeping another nutrient constant at its middle level. An elliptical contour plot implies a significant interaction between variables (Figure 3(Fig. 3)). The statistically optimal values of parameters were achieved by moving along the major and minor axes of the contour. When the Trisodium citrate kept 3.14 g, the EPS yield would decrease after increase with the content of Dipotassium hydrogen phosphate and Tween 80 increasing. When the Dipotassium hydrogen phosphate was 3.50 g and Tween 80 was 0.5 ml, the EPS yield was the highest (Figure 3a(Fig. 3)). 

When Tween 80 kept 0.58 mL, the EPS yield would increase with the content of Trisodium citrate increasing, while decrease after increase with the content of Dipotassium hydrogen phosphate increasing. When Trisodium citrate and Dipotassium hydrogen phosphate were 4.0 g and 3.60 g respectively, the EPS yield was the highest (Figure 3b(Fig. 3)). When Dipotassium hydrogen phosphate kept 3.38 g, the EPS yield would increase with the content of Trisodium citrate increasing, while decrease after increase with the content of Tween 80 increasing. When Trisodium citrate and Tween 80 were 4.0 g and 0.5 mL respectively, the EPS yield was the highest (Figure 3c(Fig. 3)). The optimum predicted value is obtained in the smallest ellipse in the contour diagram. The optimum levels of each variable were found to be Tween 80 0.6 mL, Dipotassium hydrogen phosphate 3.6 g, and Trisodium citrate 4.1 g for a predicted EPS yield of 4.02 g/L. Under the optimized fermentation parameters, the highest EPS yield reached 3.96±0.08 g/L, which had no significant difference with the predicted value of the model (4.02 g/L) (P > 0.05). It was higher than that of the control (1.05±0.06 g/L) significantly (P < 0.05). RSM used in our research is a collection of mathematical and statistical techniques for designing experiments, building models, searching optimum conditions of factors for desirable responses and evaluating the relative significance of several affecting factors even in the presence of complex interactions (Mohana et al., 2008[29]; Ruchi et al., 2008[41]; Yao et al., 2009[51]). Many articles demonstrate that RSM is effective to optimize fermentation conditions of different strains for higher EPS yields (Li et al., 2009[26]; Xiao et al., 2007[48]; Xu et al., 2010[50]). Most researches have been indicated that fermentation temperature, fermentation time and inoculum volume are the most significant influence factors in the optimization with RSM (Gao and Gu, 2007[14]; Zhao et al., 2009[53]). However, in the present study, the most significant factors in fermentation conditions optimization were Dipotassium hydrogen phosphate, Trisodium citrate and Tween 80. Tween 80 is a growth factor for *L. acidophilus* and when its concentration increases, the growth of *L. acidophilus* is stimulated*.* However, Tween 80 is also a surfactant and when it is excessive; the membrane of *L. acidophilus* will be destroyed, causing the death of *L. acidophilus*. The reason that Dipotassium hydrogen phosphate and Trisodium citrate affect the yield of EPS produced by *L. acidophilus* significantly may be that they could adjust the pH of fermentation broth as buffer agent. It is clear that pH of fermentation broth is one of the most environmental conditions that could affect the EPS production (Årsköld et al., 2007[1]; Kuntiya et al., 2010[23]; Ricciardi et al., 2002[37]). In the present study, the EPS yield was promoted by 277.14 % through optimizing the three factors with RSM.

The article "Yield improvement of exopolysaccharides by screening of the Lactobacillus acidophilus ATCC and optimization of the fermentation and extraction conditions" was published in 2016. Journal: EXCLI J.

### Screening extraction conditions with CCD design

After the variables (alcohol concentration, M/L ratio, extraction time) were identified via the single experiments (data not shown), the CCD experiment (Table 2(Tab. 2)) was operated and analyzed, which was a method of RSM applied to determine the optimal levels of selected variables (Wang et al., 2007[47]).

The equation used to explain the extraction yield of EPS produced by *L.acidophilus* initial strains is as follows [Equation 3]:

Y=-27.4+0.762X_1_+0.985X_2_-0.069X_3_-0.005X_1_^2^-0.203X_2_^2^+0.005X_3_^2^+0.001X_1_X_2_-0.003X_1_X_3_+0.014X_2_X_3_. [3]

Regression analysis showed that alcohol concentration and M/L ratio had a significant positive linear effect on the extraction yield of EPS (P < 0.01) and extraction time had a negative effect on the extraction yield of EPS. The M/L ratio had the highest impact on the extraction yield (the coefficient is 0.985) and the extraction time had the lowest impact (the coefficient is 0.069). The quadratic and interactive effects were also significant. The interactive effects of various factors on extraction ratio of EPS were presented in Figure 4(Fig. 4). The elliptical contour plot implied a significant interaction between the two variables with the rest variable at middle level. When extract time kept 24 h, the extraction ratio of EPS would increase firstly and then decrease with the ratio of M/L and concentration of ethanol increasing. Polysaccharide is not soluble in ethanol; therefore, more polysaccharide can be precipitated by increasing the concentration of ethanol moderately. On the other hand, because the ratio of M/L means the ratio of the supernatants to ethanol, it has the corresponding effect on the extraction ratio of EPS with the ethanol concentration. When the concentration of ethanol and ratio of M/L were 72.5 % and 1:3.5 respectively, the extraction ratio of EPS was the highest (Figure 4a(Fig. 4)). When the concentration of ethanol kept 70 %, the extraction ratio of EPS would increase with the ratio of M/L increasing, which further proved that the ethanol content has a significant effect on polysaccharide extraction. While the extraction ratio decreased firstly and then increase with the extraction time increasing. When the extract time and ratio of M/L were 30 h and 1:3.5 respectively, the extraction ratio of EPS was the highest (Figure 4b(Fig. 4)). When the ratio of M/L kept 1:3, the extraction ratio of EPS would increase firstly and then decrease with the concentration of ethanol increasing. However, it would firstly decrease and then increase with the extract time increasing. When the concentration of ethanol and extract time was 70 % and 30 h, the extraction ratio of EPS was highest (Figure 4c(Fig. 4)). The optimum levels of each variable were determined to be as follows: the alcohol concentration was 70 %, M/L ratio was 1:3.6, and the extraction time was 31 h. At these optimum levels, EPS extraction yield of 1.48±0.23 g/L was obtained, which had no significant difference with the predicted value (1.56 g/L) (P > 0.05). It was higher than that of the control (1.05±0.06 g/L) significantly (P < 0.05). Although there were many articles about EPS extraction of microorganism (Chen et al., 2012[9]; Gan et al., 2011[13]), while in the present study, the extraction condition was firstly optimized with CCD design. The EPS extraction yield was promoted by 48.57 % under the optimized extraction conditions. 

The article "Yield improvement of exopolysaccharides by screening of the Lactobacillus acidophilus ATCC and optimization of the fermentation and extraction conditions" was published in 2016. Journal: EXCLI J.

### Verification experiments 

The *L. acidophilus *ATCC mutant strain (No. 48) was selected to be fermented in the optimized incubators (Tween 80 0.6 mL, Dipotassium hydrogen phosphate 3.6 g, and Trisodium citrate 4.1 g), and the EPS was extracted under the optimized conditions (alcohol concentration 70 %, M/L ratio 1:3.6, extraction time 31 h). The EPS yield under the optimized conditions was 5.12 ±0.73 g/L, which was 4.88 times as much as that of the control (1.05±0.06 g/L).

## Conclusions

To gain the strains with high-yielding EPS,* L. acidophilus *ATCC initial strains were mutated by diethyl sulfate. No. 48 mutant strain was screened with the EPS yield of 2.92±0.05 g/L. To increase the EPS yield produced by *L. acidophilus *ATCC, 16 fermentation parameters, including medium compositions and culture conditions were optimized by PB design for maximal EPS yield. The three important parameters (Dipotassium hydrogen phosphate, Tween 80 and Trisodium citrate) had significant effect on EPS yield. The optimum values of these three variables were identified by RSM design. The EPS extraction conditions were optimized by CCD design to gain higher EPS extraction rate. The results indicated a novel EPS-producing strain (No. 48) from *L. acidophilus* ATCC and illustrated the optimum conditions of its EPS production and EPS extraction. Moreover, the rheology of fermentation broths was first applied to preliminary strains screen, which can greatly reduce the production cost and labour intensity. The work built up proper models to optimize the EPS fermentation and extraction conditions.

## Acknowledgements

This study was supported by the Chinese National 863 Plan (Grant No. 2006AA10Z330), the Chinese National Natural Science Fund (Grant No. 30171074), the Science Research Program of Hubei Ministry of Education (Grant No. B2014235).

The article "Yield improvement of exopolysaccharides by screening of the Lactobacillus acidophilus ATCC and optimization of the fermentation and extraction conditions" was published in 2016. Journal: EXCLI J.

## Author contributions

Proposed the theoretical frame: QL, SP, FY; Conceived and designed the experiments: QL, XH, DY, FY; Contributed reagents/materials/analysis tools: SP, FY; Wrote the paper: QL, FY; Performed the experiments: QL, DY, FY; Analyzed the data: QL, FY.

## Figures and Tables

**Table 1:** Fermentation process optimization of EPS produced by activated *L. acidophilus *ATCC*. * Experimental design and results of PB on the fermentation process optimization of EPS produced by L. acidophilus^*^.

**Table 2:** Fermentation process optimization of EPS produced by activated *L. acidophilus *ATCC*. * Experimental design and results of BBD on the fermentation process optimization of EPS produced by activated *L. acidophilus *ATCC (n=3, Mean±SEM)*.*

**Table 3:** Experimental design and results of CCD on the extraction process optimization of EPS produced by activated *L. acidophilus *ATCC (n=3, Mean±SEM).

**Table 4:** EPS yields of the 19 mutant strains and the control in MRS broth medium after incubation at 37 °C for 24 h (n=3, Mean±SEM)

**Table 5:** Fermentation process optimization of EPS produced by activated *L. acidophilus *ATCC*. *The design of the steepest ascent experiment

**Table 6:** Fermentation process optimization of EPS produced by activated *L. acidophilus *ATCC*. *The results of the steepest ascent experiment (n=3, Mean±SEM)

**Figure 1:** The viscosity of milk fermented with 54 mutant strains and the control^* ^(n=3, Mean±SEM). ^* ^No. 1 - No. 54 represented the 54 mutant strains and the No. 55 represented the control (initial strain).

**Figure 2:** Significance of 16 variables on EPS yields from activated* L. acidophilus *ATCC. (a) Represented the pareto chat rationalizing the effect of each variable on EPS yield. The standard effects of 16 variables were calculated by MINITAB 16. The average standard effect was 2.07. (b) Represented the main effect of variables on EPS yield. The slope of each variable was steeper; the influence of each variable was greater.

**Figure 3:** 2D contour plot of EPS yield for the effect of cross-interaction among Tween 80, Dipotassium hydrogen phosphate and Trisodium citrate. a: Cross-interaction between Tween 80 and Dipotassium hydrogen phosphate. Hold value: Trisodium citrate-3.14g. b: Cross-interaction between Trisodium citrate and dipotassium hydrogen phosphate. Hold value: Tween80-0.58mL. c: Cross-interaction between Trisodium citrate and Tween 80. Hold value: Dipotassium hydrogen phosphate-3.38g.

The article "Yield improvement of exopolysaccharides by screening of the Lactobacillus acidophilus ATCC and optimization of the fermentation and extraction conditions" was published in 2016. Journal: EXCLI J.

**Figure 4:** Contour plot of EPS extraction for the effect of cross-interaction among alcohol concentration, M/L ratio and extraction time. a: Cross-interaction between M/L ratio and concentration of ethanol. Hold value: extraction time 24 h. b: Cross-interaction between extraction time and M/L ratio. Hold value: alcohol concentration 70 %. c: Cross-interaction between extraction time and alcohol concentration. Hold value: M/L ratio 1:3.
